RETRACTED

# PRL/PRLR Can Promote Insulin Resistance by Activating the JAK2/STAT5 Signaling Pathway

**DOI:** 10.1155/2022/1456187

**Published:** 2022-10-04

**Authors:** Pei-yu Wang, Cong-cong Jin, Chang Liu, Zhou-jian Zhao, Hai-yan Yang

**Affiliations:** ^1^Reproductive Medicine Center, The First Affiliated Hospital of Wenzhou Medical University, Wenzhou, Zhejiang 325000, China; ^2^Zhuji Yaojiang Town Central Health Center, Shaoxing, Zhejiang 311822, China

## Abstract

**Objective:**

Although prolactin (PRL) is known to affect food intake, weight gain, and insulin resistance, its effects on lipid metabolism and underlying mechanisms remain underinvestigated. This study aimed to investigate the effects of PRL and its receptor (PRLR) on fat metabolism in regulating the JAK2/STAT5 signaling pathway.

**Methods:**

SW872 adipocytes were incubated with oleic acid to establish an insulin resistance (IR) model. Western blot was used to detect the expression of PRLR, JAK2, p-JAK2, STAT5, and p-STAT5. Triglyceride (TG) mass was detected by chemical colorimetry methods.

**Results:**

Fat droplets in the high-dose and medium-dose PRL groups were significantly higher than in the IR model group. TG mass in the cells was increased significantly compared with the model group. Compared with the control group, the expression of PRLR, p-JAK2, and p-STAT5 were significantly decreased in the IR model group when PRL was intervened for 24 h and 48 h. The expression of PRLR, p-JAK2, and p-STAT5 in the high-dose PRL intervention group increased significantly compared with the model group. The PRLR overexpressing group had significantly increased TG content and PRLR, and JAK2, p-JAK2, STAT5, and p-STAT5 levels compared with the IR model.

**Conclusion:**

PRL and PRLR are related to fat metabolism, and the PRL/PRLR signaling pathway can promote insulin resistance by activating the JAK2/STAT5 signaling pathway and increasing the deposition of TGs.

## 1. Introduction

Insulin resistance (IR) is caused by decreased biological activity of insulin in the body, including a decrease in insulin sensitivity and responsiveness. Insulin resistance has been shown to occur in the classic insulin-responsive organs such as the liver, skeletal muscle, and white adipose tissues [1–3]. It was shown to be the most important and fundamental reason for the occurrence and development of diabetes, hypertension, hyperlipidemia, and other diseases [4–6]. Presently, metabolic syndrome and type 2 diabetes have become chronic global epidemic diseases [7]. Therefore, finding ways to counter insulin resistance is a current focus of medical research.

Prolactin (PRL) is a pituitary hormone known to control the initiation and maintenance of lactation [8, 9]. However, the PRL receptor is expressed in the endometrium, prostate, islets, and adipocytes, indicating that it is also involved in various other physiological functions, including metabolism [10, 11]. Studies have shown that PRL could affect food intake, weight gain, and insulin resistance by inhibiting the production of adiponectin and IL-6 in adipose tissue [8, 12–14]. PRL can also affect the growth of pancreatic*β* cells and reduce the glucose threshold to stimulate insulin secretion [15–17], indicating that PRL has a protective effect on type 2 diabetes.

RETRACTED

The PRL receptor (PRLR) belongs to the cytokine receptor superfamily and is characterized by its ability to activate Janus kinases (JAKs) and the signal transducers and activators of transcription (STAT) transcription factors [18, 19]. In the unstimulated state, STATs were shown to localize throughout the cell, but upon stimulation, they are phosphorylated and induce their dimerization and translocation into the cell nucleus to bind to specific DNA elements known as *γ*-activated sequence-like elements (GAS) and modulate the expression of target genes [20]. The PRLR can also activate a subset of STAT proteins, including STAT1, STAT3, STAT5A, and STAT5B [21]. Although the physiological significance of STAT1 and STAT3 activation by PRL is unclear, the generation of STAT5A and STAT5B knockout mice showed that these STAT5 isoforms have essential roles in the biological actions of PRL [22, 23].

The role of PRL induction is believed to be very complex in humans as it varies based on different conditions. Thus, the exact role and underlying mechanisms of PRL on insulin resistance are yet to be fully discovered. Thus, the aim of this study was to determine the role of PRL and PRLR in lipid metabolism and the probable underlying mechanisms.

## 2. Materials and Methods

### 2.1. Cell Culture and Modeling

SW872 adipocytes were obtained from Beina Biotech Co. Ltd. They were cultured in DMEM at 37 °C with 5% CO_2_. The cells were digested and harvested, then diluted and inoculated in a 24-well plate (3 × 10^4^/well). After the cells completely adhered to the well, oleic acid (0.6 mmoL/L) [24] was added, and the cells were incubated at 37 °C for 72 h. Oil red O staining was performed to verify the modeling effects.

### 2.2. PRL Treatment

Cells were divided into five groups: control group, IR group, and different doses of PRL treatment groups (PRL-H 300 ng/mL, PRL-M 200 ng/mL, and PRL-L 100 ng/mL). The model cells were treated with 0.6 mmoL/L of oleic acid for 24 h, except for the control group. Then, the culture medium was changed, and the cells were washed twice with phosphate-buffered saline (PBS) to remove the oleic acid on the cell surface. To evaluate whether the effect of PRL was related to the duration of treatment, they were treated with different doses of PRL for 24 h and 48 h, respectively.

RETRACTED

### 2.3. Cell Transfection

Vectors for the overexpression and shRNA targeting of PRLR using lentiviral gene transfer were constructed by GenePharma (Shanghai, China). SW872 adipocytes were seeded at 5 × 10^5^ cells per well in 6-well plates. Transfection was conducted when the cell density reached 70%, followed by transfection of the overexpressed PRLR plasmid using Lipofectamine 3000 (Invitrogen) according to the manufacturer's instructions. After transfection of 48 hours, the cells were harvested for further experiments.

### 2.4. Western Blot

Total proteins were extracted from different groups. A BCA kit was used to determine the protein concentration, and the proteins were separated by 12% SDS-PAGE. They were electrotransferred to a PVDF membrane and rinsed for 15 min with TBS. The membrane was blocked, followed by the addition of appropriate dilution of primary antibodies (PRLR: 1 : 1000, cat. no.#13552; JAK2: 1 : 1000, cat. no.#3230; p-JAK2 Tyr1007/1008: 1 : 1000, cat. no.#3776; STAT5: 1 : 1000, cat. no.#94205; p-STAT5 Tyr694: 1 : 1000, cat. no. #9359; amd GAPDH: 1 : 1000, cat. no. #5174) purchased from Cell Signaling Technology, and incubation at 4 °C overnight. The membrane was rinsed and then incubated with a secondary antibody at room temperature for 2 h. Then, bands were determined by using the enhanced chemiluminescence kit. Image J software was used to observe and analyze them.

### 2.5. Oil Red O Stain

Lipid droplets were stained with Oil red O (ORO) obtained from Sigma. The cells were rinsed three times in PBS and fixed in 10% (v/v) paraformaldehyde for 15 min and washed with 60% isopropanol for 20 s followed by Oil red O staining for 15 min at room temperature. Then, they were rinsed with 60% isopropanol, destained, and stained with hematoxylin for 1 min. They were then rinsed with 60% alcohol for 10 s, after which the blue returning liquid was added for 15 s, rinsed with water, and sealed with glycerin gelatin. Images were collected using an inverted microscope (Olympus, IX-70, Tokyo, Japan).

### 2.6. Determination of Total Triglyceride (TG)

The content of TG in the cell supernatant and intracellular was determined using a TG detection kit (Applygen Technologies; Beijing, China) according to the manufacturer's instructions. In brief, cells were seeded at 2 × 10^3^ cells/cm^2^ in 6-well plates. Cells were harvested at indicated time points after corresponding processing, rinsed three times with PBS, scraped off the plates, and lysed with RIPA lysis buffer (Beyotime; Shanghai, China) for 30 min. The triglyceride content of the cells was measured at 490 nm. Total protein concentration was estimated by the BCA method (Beyotime) according to the manufacturer's instructions. The total amount of TG in the cells was expressed by the amount of TG in each milligram of total cell protein.

RETRACTED

### 2.7. Statistical Analysis

The data were analyzed using the Graphpad Prism7 software. All data are presented as *mean* ± *standard* *deviation* (SD). The differences among groups were evaluated by one-way ANOVA. *P* < 0.05 was used to indicate statistical significance.

## 3. Results

### 3.1. Identification of Mature Adipocytes by Oil Red O Staining

Oil red O staining was used to identify whether SW872 preadipocytes were induced into mature adipocytes (Figure 1). The results showed that compared with preadipocytes, the number of red stained granules in the induced cells increased, indicating lipid accumulation and that the induction was successful.

### 3.2. Effects of Different Doses of PRL on Lipid in IR Cells

To explore the effect of different doses of PRL on the lipid in IR cells, Oil red O staining was used to detect the lipid content in each group. The selection of the three dosages (300 ng/mL, 200 ng/mL, and 100 ng/mL) was according to our preliminary experiment which proved they are effective and have no toxicity in cells. The results (Figures 2(a)–2(b)) showed that the lipid content in the IR model group was significantly higher than in the control group (*P* < 0.05). The lipid content in the high and middle-dose PRL group was further increased than the IR model group (*P* < 0.05). Further, there was no significant decrease in lipid content after low-dose PRL treatment (*P* > 0.05). The lipid content in the high and middle-dose PRL group was significantly higher than in the low-dose PRL group (*P* < 0.05).

### 3.3. Effect of Different Doses of PRL on TG Content in IR Cells

Here, we investigated how different doses of PRL would affect the content of TG in the IR cells. As shown in Figure 3, in the cell supernatant, the TG content in the IR model group was significantly higher than in the control group (*P* < 0.05). The TG content decreased with the increase of PRL dosage. The TG content in IR model cells was also significantly higher than in the control group (*P* < 0.05). At 48 h, there was no significant difference in TG content between the high-dose group and the model group, but the TG content was found to be significantly increased in the middle dose group and significantly decreased in the low-dose group (*P* < 0.05).

### 3.4. Effects of Different Doses of PRL on PRLR and JAK2/STAT5 Signaling Pathway in IR Cells

Here, we investigated the effect of the different doses of PRL on the JAK2/STAT5 signaling pathway. At 24 h, the expressions of PRLR, JAK2, p-JAK2, STAT5, and p-STAT5 in the IR model group were significantly decreased compared with that of the control group. The expression levels of PRLR, JAK2, p-JAK2, STAT5, and p-STAT5 were significantly increased in the high-dose PRL group compared with the model group (Figure 4(a), *P* < 0.05). At 48 h, the expressions of PRLR, p-JAK2, and p-STAT5 were significantly decreased, while JAK2 expression was significantly increased in the IR model group compared with the control group. In addition, the expression levels of PRLR, p-JAK2, and p-STAT5 were significantly increased, while JAK2 expression was significantly decreased in the high-dose PRL group compared with that of the model group (Figure 4(b), *P* < 0.05).

RETRACTED

### 3.5. Effect of PRLR Overexpression on Intracellular TG Content in IR Cells

To further confirm the relationship between PRLR and IR, we treated IR cells with overexpression of PRLR. As shown in Figure 5(a), the expression of PRLR was significantly increased compared with the empty vector and control group, which suggests the successful construction of the PRLR overexpression vector. Next, we determined the TG content to explore the effect of overexpressed PRLR. The TG content in the IR model group increased significantly compared with the control group (*P* < 0.05), while the TG content in the PRLR overexpression group was further significantly increased than the IR model group (Figure 5(b), *P* < 0.05).

### 3.6. Effects of PRLR Overexpression on PRLR and JAK2/STAT5 Signaling Pathways in IR Cells

To further confirm PRLR takes effect through JAK2/STAT5 signaling pathways, we overexpressed PRLR and detected related protein. The expressions of PRLR, JAK2, p-JAK2, STAT5, and p-STAT5 in the IR model group were significantly decreased compared with the control group. The expression levels of PRLR, JAK2, p-JAK2, STAT5, and p-STAT5 were significantly increased in the PRLR overexpressed group compared with the model group (Figure 5(c), *P* < 0.05).

## 4. Discussion

Insulin resistance is one of the common causes of metabolic syndrome, including coronary heart disease and diabetes. It is considered as the “common soil” of metabolic syndrome. The mechanism of IR has not been fully elucidated. The high cost, long-term, and difficult operation of the research restrict the development of a large number of experiments on the mechanism *in vivo* in humans and animals. Therefore, the establishment of the IR cell model becomes a fast and effective method to study the mechanism of IR.

RETRACTED

Many studies have shown that adipose tissue is not only a passive energy storage organ but also an endocrine organ that can secrete hormones. Abnormal proliferation and differentiation of adipocytes can lead to excessive adipose tissue accumulation, leading to obesity and IR [10, 11]. Oleic acid is a monounsaturated fatty acid. It was proved that oleic acid could promote the expression of PPAR*γ*, C/EBP*α*, and lipoprotein lipase (LPL) in adipocytes, which indicated that oleic acid could be used as an inducer of adipocyte differentiation [12]. SW872 preadipocytes are human-derived adipocyte lines, and oleic acid can successfully induce SW872 preadipocytes to differentiate into mature adipocytes [13]. This study was consistent with it. We found that after 72 hours of oleic acid induced the differentiation of SW872 preadipocytes, there were abundant lipid droplets in the cytoplasm, which proved that the induction was successful.

PRL was identified as a metabolic hormone [15]. PRL can regulate the secretion of adipokines such as adiponectin and leptin [16, 17]. The report showed the inhibitory effect of PRL on lipid synthesis in the liver of female rats [25]. In this study, we found that PRL treatment and overexpression of PRLR significantly increased TG content in SW872 cells induced by oleic acid and found that a higher concentration of PRL was associated with a higher increase in TG content. However, Zhang et al. proposed that PRL of 20 ng/ml (near the normal range of the human body) had beneficial effects on liver lipid metabolism, but PRL of high concentration (> 100 ng/ml) may not have beneficial effects on liver lipid metabolism [26]. Prolactin activation of the long form of its cognate receptor causes increased visceral fat and decreased fatty acid oxidation [27]. PRL has different or opposite effects on different animals and tissues, which may be related to the diversity of PRLR receptors and the different regulatory roles of different types of PRLR receptors. In this study, PRL/PRLR can promote IR and accelerate lipid droplet deposition.

The JAK/STAT signaling pathway played an important role in lipid metabolism [28–30]. Some studies showed that STAT5 activation improved liver fat deposition by inhibiting CD36 in mice [31, 32]. However, Corbit et al. found that JAK2 expressed in fat and liver had opposite effects on lipid accumulation [33]. Previous studies also showed that STAT5A and STAT5B promoted adipogenesis and the accumulation of fat droplets in adipocytes [34, 35]. In this study, a high concentration of PRL or PRLR overexpression treatment could significantly upregulate the protein expression levels of p-JAK2 and p-STAT5 in IR adipocytes, which indicated that PRL/PRLR promoted fat deposition in adipocytes by activating JAK2/STAT5 pathway, leading to an increase in TG.

RETRACTED

## 5. Conclusions

In conclusion, activation of the PRL/PRLR signaling pathway could activate JAK2/STAT5 phosphorylation and increase TG deposition. However, the effects of low concentration PRL on lipid metabolism need to be further explored. Moreover, the therapeutic effect of the PRL/PRLR signaling pathway on insulin resistance-related diseases needs more relevant experimental evidence.

## Figures and Tables

**Figure 1:** Oil red O staining results. Representative images of Oil red O stained lipid droplets (red) and hematoxylin-stained nuclei (blue) in SW872 adipocytes. There is no lipid accumulation in SW872 preadipocytes, while SW872 mature adipocytes have a substantial lipid accumulation (the red arrow) in the cytoplasm of the cells and have some large lipid vacuoles (the black arrow) in fully differentiated adipocytes.

**Figure 2:** Effects of different doses of PRL on lipid in IR cells. (a) Oil red O staining in SW872 adipocytes allowed to analyze the differences of lipid accumulation in the cytoplasm of the cells in different groups. The lipid accumulation (see the arrow). (b) Statistical analysis of the lipid content in different groups. ∗*P* < 0.05, *vs*. Control group; #*P* < 0.05*vs*. IR group. Abbreviations: PRL: prolactin; IR: insulin resistance; PRL-M: PRL middle dose; PRL-L: PRL low dose; PRL-M: PRL middle dose; PRL-H: PRL high dose.

**Figure 3:** Effects of different doses of PRL on the triglyceride content. (a) Determination of the content of TG in cell supernatant of different groups after 24 h PRL treatment and 48 h PRL treatment. (b) Determination of the content of TG in intracellular of different groups after 24 h PRL treatment and 48 h PRL treatment. ∗*P* < 0.05*vs*. Control; #*P* < 0.05*vs*. IR model group. Abbreviations: PRL: prolactin; IR: insulin resistance; PRL-M: PRL middle dose; PRL-L: PRL low dose; PRL-M: PRL middle dose; PRL-H: PRL high dose.

**Figure 4:** Effects of different doses of PRL on PRLR and JAK2/STAT5 signaling pathway in IR Cells. (a) Western blot detect the expressions of PRLR, JAK2, p-JAK2, STAT5, and p-STAT5 of different groups after PRL treatment for 24 h. (b) Western blot detect the expressions of PRLR, JAK2, p-JAK2, STAT5, and p-STAT5 of different groups after PRL treatment for 48 h. ∗*P* < 0.05*vs*. Control; #*P* < 0.05*vs*. IR model group. Abbreviations: PRL: prolactin; IR: insulin resistance; PRL-M: PRL middle dose; PRL-L: PRL low dose; PRL-M: PRL middle dose; PRL-H: PRL high dose.

**Figure 5:** Effects of PRLR overexpression on intracellular triglyceride content through JAK2/STAT5 signaling pathways in IR cells. (a) Western blot detect the expression of PRLR in the control group, empty vector and overexpression PRLR group. (b) The TG content was detected in the control group, IR group, IR + PRLR NC group, and IR + PRLR group. (c) Western blot detect the expressions of PRLR, JAK2, p-JAK2, STAT5, and p-STAT5 of different groups. ∗*P* < 0.05*vs*. Control; #*P* < 0.05*vs*. IR model group. Abbreviations: PRLR: prolactin receptor; IR: insulin resistance; NC: normal control.

RETRACTED

## Data Availability

The datasets during and/or analyzed during the current study are available from the corresponding author on reasonable request.
